The article "Investigation of the Ordered Structure in Partially Melted Isotactic Polypropylene" was retracted in 2023. Reasons: no approval from the institution; copyright claims.

# Investigation of the Ordered Structure in Partially Melted Isotactic Polypropylene

**DOI:** 10.3390/polym13193354

**Published:** 2021-09-30

**Authors:** Junfang Shen, Derong Zhu, Junchao An, Zhiyu Min, Jingbo Chen

**Affiliations:** 1 School of Materials Science and Engineering, Luoyang Institute of Science and Technology, Luoyang 471023, China; shen8009@126.com (J.S.); ajc_1979@163.com (J.A.); 2 Henan Intelligent Manufacturing Engineering Technology Research Center for Building Profile, Luoyang 471023, China; 3 School of Intelligent Manufacturing, Luoyang Institute of Science and Technology, Luoyang 471023, China; 4 School of Materials Science and Engineering, Zhengzhou University, Zhengzhou 450001, China; chenjb@zzu.edu.cn

**Keywords:** ordered structure, partial melting, isotactic polypropylene, crystallization

## Abstract

The ordered structure of partially melted isotactic polypropylene (iPP) was investigated using polarized optical microscopy (POM) and small-/wide-angle X-ray scattering (SAXS/WAXS) measurements. The crystalline morphology was first examined by means of pulling a glass fiber through the iPP melt, which was generated by partially melting a preformed spherulite. The results from the POM experiments indicated that, even at a minimal pulling rate, the surviving ordered structure could also relocate along the direction of fiber pulling and grow into cylindrites eventually. In addition, during the quiescent crystallization from the partially melted sample, which had the same thermal history of fiber-pulling experiments, the obvious memory effect of melt was also observed from the results of X-ray experiments. Moreover, the SAXS profile derived from the partially melted iPP at 170 °C was fitted by the theory of scattering amplitude with the cylindrical form factor. The fit result implied that the surviving ordered structure is of cylindrical nanocrystals with a diameter *D* ≈ 30 ± 3 nm and height *h* ≈ 45 ± 3 nm, which can significantly influence the crystallization morphology and kinetics during the subsequent crystallization process.

## 1. Introduction

Crystallization is a rearrangement process of polymer chains from a disordered to an ordered state [1]. For chain-folded polymers, the formation of lamellae structure depends on the crystallization kinetics upon cooling [2,3,4]. As we know, crystalline structures are in thermal disequilibrium. Therefore, these structures are classed as metastable states in thermodynamics, with a significant degree of imperfections [1,5,6]. During the later heating process, the melting behavior is strongly influenced by the metastable structure that has formed previously.

For semi-crystallization polymers, melting behavior can be highly complicated. It covers a certain temperature range that is ascribed to the thickness distribution of the lamellae [7,8,9,10,11,12]. According to the Gibbs-Thomson equation, a thicker lamella is more stable and has a higher melting point than those that are thinner [13,14]. At the same time, because of the effect of melt-recrystallization, the lamella is thickening during heating until melting [13,15,16,17,18,19,20]. Based on abundant experiments by means of small-angle X-ray scattering (SAXS) measurements [21,22,23], the melting behavior of semi-crystallization polymers was depicted with a melting line and recrystallization line by Strobl and co-workers. The melting line denoted the linear relationship between the inversed lamellar thickness (*d_c_*^−1^) and melting temperature (*T_m_*), while the recrystallization line showed a continuous thickening process upon heating. This melting behavior was further confirmed by Men [24,25,26]. All the melting behaviors investigated by them are based on the existence of a periodic lamellar structure. However, the nature of the surviving ordered structure after the periodic lamellar structure’s disappearance was not mentioned.

The article "Investigation of the Ordered Structure in Partially Melted Isotactic Polypropylene" was retracted in 2023. Reasons: no approval from the institution; copyright claims.

On the other hand, when a crystalline polymer is melted between the nominal melting point (*T_m_*) and equilibrium melting point (*T*^0^*_m_*), the surviving ordered structures in the melt will significantly influence its following crystallization. This phenomenon is often referred to as a self-nucleation or melt memory effect [27,28,29,30,31,32] and the surviving structure was often called the precursor. For its fundamental scientific and industrial possibilities, the melt memory effect has received a great deal of attention since it was first revealed in the 1960s [33]. Many previous reports were focused on the effect of precursors on crystallization [34,35]. However, the nature and origin of the precursors that survived in the partial melting of polymers were seldom reported. On the basis of research about melting kinetics in polymers by Rastogi [36,37,38], a multistage melting process was observed during heating. In the low melting-temperature region, melting occurred through the detachment of chain stems from the lamellar surface, whereas in the high melting-temperature region, melting led to a breakdown of the lamellar framework. Luo et al. [39] researched the melting and growth of polymer crystals during heating with molecular dynamics simulations and suggested that infusible microcrystalline domains at high temperatures could be the seeds of subsequent nucleation events. In addition, some researchers directed their attention to the shape and size of precursors in the early stages of crystallization. Cheng et al. studied primary nucleation in the polymer crystallization of poly(ethylene oxide) and considered that the primary nuclei should be rod-like [28]. Moreover, the size of this rod-like precursor can be estimated by a Guinier plot with SAXS data. Han et al. acquired the average radius of gyration of critical nuclei in the first several minutes of the nucleation process in the isothermal crystallization of polyethylene [40]. In previous works [41,42], the form factor was employed to analyze the size and shape of the ordered structure that existed in the partial melting of iPP after the periodic lamellar structure was melted. It was suggested that the nanocrystals were produced by controlling the melt structure in partially melted iPP.

The article "Investigation of the Ordered Structure in Partially Melted Isotactic Polypropylene" was retracted in 2023. Reasons: no approval from the institution; copyright claims.

In this study, the surviving ordered structure in partially melted iPP was investigated by polarized optical microscopy (POM) and small-/wide-angle X-ray scattering (SAXS/WAXS) measurements. Firstly, the relocation of the surviving ordered structure was examined by pulling a glass fiber through the partially melted iPP. POM was employed to observe the evolution of crystalline morphologies during the fiber-pulling experiments. Subsequently, the quiescent crystallization from the partially melted sample, which had the same thermal history as fiber-pulling experiments, was investigated by means of in situ SAXS/WAXS measurements. Moreover, in order to probe the origin of the ordered structure in the partially melted iPP, a corresponding melting experiment was conducted.

## 2. Materials and Methods

### 2.1. Material and Sample Preparation

The isotactic polypropylene (iPP), F401 (*M_n_* = 83,000, *M_w_* = 315,000, *MWD* = 3.79), used in this work was provided by the Yangzi Petroleum Chemical Corp., Nanjing, China. A melt flow index of 3.0 g/10 min was measured with a load of 2.16 kg at 230 °C. The nominal melting temperature (*T_m_*) was about 166 °C, measured by DSC at 10 °C/min. Two types of iPP films with a thickness of ca. 1 mm (for X-ray measurements) and 30 μm (for fiber-pulling experiments) were prepared by compression molding at 210 °C for 10 min and subsequently quenched to room temperature in air. The glass fiber (GF) with a diameter of ca. 14 μm was provided by Henan ZhengTong Chemical Co. Ltd., Zhengzhou, China. In order to remove the possible impurity on the fiber surface, the fiber was rinsed for 30 min with acetone and then dried at 80 °C for 8 h in a vacuum oven.

For the fiber-pulling experiment, a single fiber was sandwiched between two thin iPP films and confined between two cover glasses. A homemade fiber-pulling device equipped with a hot stage was employed to control the pulling rate at a constant linear velocity.

The article "Investigation of the Ordered Structure in Partially Melted Isotactic Polypropylene" was retracted in 2023. Reasons: no approval from the institution; copyright claims.

### 2.2. Polarized Optical Microscopy (POM)

To observe the evolution of morphology and structure during the fiber-pulling experiments, Olympus BX-51 (Olympus, Tokyo, Japan) polarized optical microscopy (POM) was used in this study. The experimental protocol is shown in Figure 1. The sandwich sample was first heated to 210 °C for 10 min to erase the previous thermal and mechanical history. Subsequently, it was cooled down to 135 °C and kept at this temperature for 30 min. After a careful choice, a sample with preformed spherulite surrounding the fiber was selected as a candidate. Then, the temperature was increased to the testing temperature (*T_s_* = 170 °C), which was below the equilibrium melting point (*T*^0^*_m_*). After equilibration at *T_s_* for 10 min, the glass fiber was pulled through the melt at a chosen linear velocity (*V_s_*) over a distance by the fiber-pulling device. After the cessation of pulling, the sample was cooled down to 135 °C for isothermal crystallization again. The heating and cooling temperature rates were 20 °C/min during the entire experiment. All the optical micrographs shown in this article were taken under crossed polarized light.

### 2.3. X-ray Measurements

The simultaneous SAXS/WAXS investigation was performed with a Nano-inXider (λ = 0.154 nm, Xenocs, France). The X-ray source was a 40-μm-microfocus sealed tube with a copper anode and a total power of 30 W. Two “Pilatus 3” detectors (pixel size = 172 × 172 μm) were employed to detect the SAXS (487 pixels × 390 pixels) and WAXS (487 pixels × 195 pixels) signal simultaneously. The SAXS detector was positioned typically 938 mm from the sample, whereas the WAXS detector was placed 79 mm from the sample. A high temperature-controlling sample holder, Linkam HFSX350 (Tadworth, UK), controlled by a T95 system controller, was installed in the Nano-inXider. The same thermal protocol was chosen for the small-/wide-angle X-ray scattering (SAXS/WAXS) experiment, as shown in Figure 1.

### 2.4. SAXS and WAXS Data Analysis

#### 2.4.1. SAXS Data Analysis

One-dimensional SAXS profiles were derived from the two-dimension images using the Foxtrot 3.2.7 software (Xenocs, Grenoble, France). In order to establish more detailed structural information of the sample, such as lamellar thickness (*d_c_*) and the long period (*L*), the one-dimensional electron density correlation function *K(z)* was employed to analyze the SAXS data as follows:

(1) $$K(z)=\frac{\int_{0}^{\infty }I(q)q^{2}\cos(qz)dq}{\int_{0}^{\infty }I(q)q^{2}dq}$$

where the scattering vector, q=4πsinθ/λ and *z* is the real space length along the lamellar stack. The crystalline long period (*d_ac_*) can be regarded as the abscissa value of the first maximum in the *K(z)* curve; the average thickness of the stack lamellae (*d_c_*) or amorphous layers (*d_a_*) can be derived from the abscissa of the intersection of the baseline across the first minimum of *K(z)* and the linear regression in the self-correlation triangle [42].

The article "Investigation of the Ordered Structure in Partially Melted Isotactic Polypropylene" was retracted in 2023. Reasons: no approval from the institution; copyright claims.

The relative SAXS invariant, *Q*, which can characterize the structural development of the iPP sample, can be defined as:

(2) $$Q=\int_{q_{1}}^{q_{2}}I(q)q^{2}dq$$

The finite *q* range from the experimental SAXS data was selected between *q*_1_ = 0.1 nm^−1^, taken from the first reliable data point, and *q*_2_ = 2 nm^−1^, given as the profile of *I(q)q*^2^ against *q* becoming constant.

According to previous work [41,42], it was considered that the ordered structures within melts were nanocrystals with random orientation after the lamellar structure disappeared. In order to investigate the size information of nanocrystals, the SAXS profile of a structured melt can be fitted by the theory of scattering amplitude for cylinders. The theory of scattering amplitude,$\bar{\varphi }(q)$, for a cylinder is given by:

(3) $$\varphi (q)={\left(2v\frac{\sin(qh\cos\theta /2)J_{1}(qr_{c}\sin\theta )}{(qh\cos\theta /2)qr_{c}\sin\theta }\right)}^{2}$$

Here, v denote the volume of the cylinder, while *h* and *r_c_* are the mean length and radius of the cylinder. θ is the angle between the scattering vector $\vec{q}$ and the cylinder axis. *J*_1_ is the first-order Bessel function.

#### 2.4.2. WAXS Data Analysis

One-dimensional WAXS profiles were also derived from the two-dimensional images with the Foxtrot 3.2.7 software of the Nano-inXider. The mass fraction of crystalline phase, *X_c_*, can be obtained from the following equation [43]:

(4) $$X_{c}=\frac{A_{c}}{A_{c}+A_{a}}\times 100\%$$

where *A_C_* represents the WAXS integrated intensities under crystalline peaks and *A_a_* is the WAXS integrated intensities under an amorphous halo peak.

## 3. Results and Discussion

Figure 2 showed the selected optical micrographs of crystalline morphology and structure obtained at different stages during the fiber-pulling experiment. In Figure 2a, the selected spherulite, penetrated through the center by a single fiber, was observed after isothermal crystallization at 135 °C for 30 min, with a diameter of ca. 160 μm. When the temperature was increased up to 170 °C and kept for 10 min, the birefringence disappeared completely. The zone where the spherulite was located previously was regarded as the structured melt zone in this work and was circled by a dashed line, as shown in Figure 2b. Then, a shear flow was generated by the fiber pulling at 62.5 μm/s over 250 μm along the direction marked in Figure 2b. Subsequently, the sample was cooled down to 135 °C again for isothermal crystallization. As shown in Figure 2c, the spherulite recovered in the previous location quickly. It should be noted that the fiber, of 250 μm in length, that was pulled out from the structured melt zone at 62.5 μm/s was covered with small crystals. On the other hand, no observed crystals were found on the fiber that was pulled out from outside the structured melt zone (denoted as the supercooled melt zone in this work). After isothermal crystallization at 135 °C for 15 min, cylindrites with a length of 250 μm were observed on the fiber, as shown in Figure 2d. At the same time, only a few isolated spherulites were found along the fiber that was pulled out from the supercooled melt zone. In addition, the recovered spherulite in the original zone was optically positive, as discussed by Yan [44].

The article "Investigation of the Ordered Structure in Partially Melted Isotactic Polypropylene" was retracted in 2023. Reasons: no approval from the institution; copyright claims.

According to the previous report by Varga [45,46], when the fiber was pulled through a polymer melt, the whole fiber was surrounded by cylindrites during the subsequent isothermal crystallization. However, in our fiber-pulling experiment, the cylindrites were observed only on the fiber surface that was pulled out from the structured melt zone. Two reasons were considered for this result. One was that the fiber-pulling rate employed in our experiment was very low and could not induce the formation of stable nucleation at 170 °C for the supercooled melt. The other, maybe the most important one, was that the surviving structure after partial melting in the structured melt could be relocated along the fiber-pulling direction even under such a low pulling rate and grew eventually into cylindrites as nucleation precursors.

In order to investigate the effect of pulling rate on the morphology and structure during the isothermal crystallization after fiber pulling at 170 °C, analogous fiber-pulling experiments were conducted using different fiber-pulling rates. The results are shown in Figure 3.

After isothermal crystallization at 135 °C for *t_c2_* = 15 min, the cylindrites were also observed on the other three fiber surfaces that were pulled out from the structured melt zone at a pulling rate of 12.5, 180 and 625 μm/s, just like at 62.5 μm/s in Figure 3b. It is further confirmed that the survived ordered structure after partial melting can be relocated along the fiber-pulling direction at different shear conditions. However, it should be pointed out that there were two differences in the cylindrites that were produced from the structured melt. Firstly, with an increase in pulling rate, the produced cylindrites looked denser. It is easy to understand that the nuclei, which grew into cylindrites, consist of two parts: one was from the surviving ordered structure and the other was formed by shear, induced by the higher pulling rate. With the increase in pulling rate, more and more shear-induced nuclei were generated. As a result, the total number of crystal nuclei increased. Secondly, the number of β-form crystals with the brightest part in the cylindrites also increased with an increase in the fiber-pulling rate. This can be attributed to the development of a number of oriented α-form crystals in the melt [47].

The article "Investigation of the Ordered Structure in Partially Melted Isotactic Polypropylene" was retracted in 2023. Reasons: no approval from the institution; copyright claims.

In addition, obvious differences were also observed in the crystalline morphology and structure that were generated on the fiber surface that was pulled out from the supercooled melt zone at different pulling rates. At the low pulling rate of 12.5μm/s, no crystals were observed in the supercooled melt zone, while cylindrites had been clearly observed in the structured melt zone at the same pulling rate. That is because the shear flow generated by fiber-pulling at 12.5 μm/s for 20 s was too weak to produce stable nuclei in the supercooled melt. With the increase in fiber-pulling rates, more and more crystals were observed on the fiber surface that was pulled out from the supercooled melt zone. Even when the pulling rate reached 625 μm/s, almost the same cylindrites were observed as were produced from the structured melt.

All the above results indicated that the surviving ordered structure located near the surface of the fiber can relocate by means of fiber-pulling, even at very low pulling rates. Furthermore, in order to study the mobility of the ordered structure under shear flow, three other analogous experiments were conducted with different pulling distances, at the same pulling rate of 12.5 μm/s. The results are shown in Figure 4. Whether at lower (125 μm, as shown in Figure 4a) or higher (500 μm and 750 μm, as shown in Figure 4c,d) pulling distances, the surviving ordered structure could also be “pulled” out and developed into cylindrites around the fiber surfaces. It indicated that there were plenty of ordered structures surviving in the structured melt zone after partial melting at 170 °C.

The optical microscopy results indicated that abundant ordered structures were in the partially melted iPP and can strongly influence the subsequent crystallization morphology. In order to study the structural evolution of iPP during the cooling process from both structured and supercooled melts, X-ray measurements were performed in situ. Partially melted iPP was prepared with the same thermal conditions as shown in Figure 1. To contrast the effect of different melt structures on crystallization, a supercooled melt was also prepared (the iPP sample was heated to 210 °C at 30 °C/min, firstly by Linkam HFSX350; then it was held there for 10 min to erase the former thermal and mechanical history; this was followed by cooling to 170 °C at 20 °C/min). The results are shown in Figure 5.

The article "Investigation of the Ordered Structure in Partially Melted Isotactic Polypropylene" was retracted in 2023. Reasons: no approval from the institution; copyright claims.

Obvious differences were found in the SAXS profiles obtained from structured and supercooled melts. In Figure 5a, with the temperature decrease, the scattering intensity continuously increased for the structured melt. This can be understood straightforwardly. The surviving ordered structure after partial melting can provide a suitable substrate for iPP chains and then reduce the nucleation barrier [48]. Therefore, secondary nucleation or growth could start quickly. As shown in the inset of Figure 5a, the characteristic diffraction peaks caused by the crystal cell structure were detected clearly, and the crystallinity derived from the WAXS data had been over 30% when the sample was cooled down to 135 °C again. In comparison, until the temperature decreased to 135 °C, the scattering intensity was still kept at the same level as the supercooled melt, and no characteristic diffraction peaks can be detected from the supercooled melt, as shown in Figure 5b. Obviously, for the supercooled melt, the melt structure of iPP was in a disordered state and the nucleation barrier had not been overcome. Thus, the crystallization process was still in its primary nucleation stage. The evolution of the relative SAXS invariant *Q* can be used to follow the development of the crystalline structure during the cooling process. As shown in Figure 5c, for the structured melt, a constant increase in the relative invariant *Q* was found until 147 °C. Below this temperature, the increase rate of *Q* rose suddenly. This increase in *Q* can be attributed to the rapid development of the crystalline structure and indicated that the crystallization process had changed into the crystal growth stage. This result coincided with the evolution of crystallinity derived from the WAXS data for the structured melt, which is shown in Figure 5d. In contrast, the SAXS invariant *Q* and WAXS crystallinity remained unchanged in the supercooled melt. It can, therefore, be inferred that nucleation has not been completed for the supercooled melt upon cooling to 135 °C. When the samples were cooled down to 135 °C for isothermal crystallization again, a great difference was found between the evolution of the relative invariant *Q* and crystallinity derived from the structured and supercooled melt respectively, as shown in the inset of Figure 5c,d. Thus, a great memory effect had appeared for the structured melt.

The article "Investigation of the Ordered Structure in Partially Melted Isotactic Polypropylene" was retracted in 2023. Reasons: no approval from the institution; copyright claims.

The surviving ordered structure in partially melted iPP can strongly influence the morphology and structure of subsequent crystallization. Then, a question arises: what is the nature of such a surviving ordered structure? In order to answer this question, the partial melting process that produced the ordered structure was also investigated by in situ SAXS and WAXS measurements as follows.

Some selected SAXS profiles and their corresponding WAXS profiles, which were collected during the partial melting process, are shown in Figure 6a,b respectively. Just like in many previous reports [49,50], the position of the scattering peak moved to the lower *q* region with the increasing temperature. Meanwhile, the characteristic diffraction peaks gradually weakened during the melting process. The evolution of *K(z)*, lamellar thickness (*d_c_*) and the long period (*d_ac_*) during the melting process is shown in Figure 6c. With the increasing temperature, *d_c_* increased from 14 nm up to 32 nm. It should be noted that the *d_c_* increased slowly until the temperature increased in the vicinity of 160 °C. Thereafter, *d_c_* quickly increased to the maximum, which was the last value derived from the *K(z)* profile at 169 °C. During the early stage of heating, the increase in *d_c_* was attributed to the recrystallization, leading to the lamellae becoming gradually thicker and more perfect. Subsequently, during the later stages of heating, the imperfect and thinner lamellae melted quickly when the temperature was getting closer to the melting point of iPP, while the thickest and most stable parts of the lamellae were preserved [42]. As we know, *d_c_* was the average thickness of the lamellae, which was derived from *K(z)*. That is to say, the rapid increase in *d_c_* was attributed to the melting of unstable lamellae during the later stages of the heating process. Subsequently, as the temperature increased up to 170 °C, the periodic structure disappeared, accompanied by the melting of the remaining lamellar structure. In comparison, the crystallinity derived from the corresponding WAXS data, *X_c_*, decreased gradually with the increase in temperature, which is shown in Figure 6d.

Although the periodic structure disappeared at 170 °C, there were plenty of ordered structures that survived in the partially melted iPP, which has been confirmed by fiber-pulling experiments. As discussed in previous research [42], the surviving ordered structure consisted of nanocrystals that originated from the most stable and thickest parts of the lamellae in the partially melting iPP. Analogously, the experimental scattering intensity collected at 170 °C after periodic structure disappeared, *I(q)*, can be fitted with a form factor of polydisperse cylinders. The best fit result is shown in Figure 7. The following values were obtained from such fitting: a diameter of *D* ≈ 30 ± 3 nm and a height of *h* ≈ 45 ± 3 nm.

The article "Investigation of the Ordered Structure in Partially Melted Isotactic Polypropylene" was retracted in 2023. Reasons: no approval from the institution; copyright claims.

## 4. Conclusions

In this work, the ordered structure in partially melted iPP was investigated by in situ POM and SAXS/WAXS measurements. Some conclusions are summarized as follows:

(1) By means of pulling the partially melted iPP with a glass fiber, we observed that the ordered structure that was generated from melting a preformed spherulite at 170 °C can be relocated along the direction of fiber pulling and eventually grow, even at minimal pulling rates. When we increased the pulling rate, the cylindrites produced from the structured melt became denser, which can be attributed to synergism between shear-induced crystallization and the relocation of surviving ordered structures in the partially melted iPP.

(2) According to the experimental results of quiescent crystallization, it can be concluded that there was a remarkable melt memory effect in the partially melted iPP.

(3) Based on the X-ray experimental results, it can be concluded that the surviving ordered structure is of nanocrystals with a diameter of 30 ± 3 nm and a height of 45 ± 3 nm, which can significantly influence crystallization kinetics during the subsequent crystallization process.

## Figures and Tables

**Figure 1:** Schematic diagram shows the thermo-mechanical protocol in the experiment.

**Figure 2:** The selected optical micrographs obtained at different fiber-pulling experimental stages. (**a**) *t_c1_* = 30 min, *T_c_* = 135 °C; (**b**) *t_s_* = 10 min, *T_s_* = 170 °C; (**c**) *t_c2_* = 2 min, *T_c_* = 135 °C; (**d**) *t_c2_* = 15 min, *T_c_* = 135 °C. The pulling rate and distance were 62.5 μm/s and 250 μm, respectively.

**Figure 3:** The selected optical micrographs obtained at *t_c2_* = 15 min after fiber pulling with different pulling rates at 170 °C: (**a**) 12.5 μm/s; (**b**) 62.5 μm/s; (**c**) 180 μm/s; (**d**) 625 μm/s. The fiber-pulling distance was 250 μm and the same pulling direction was marked in (**b**).

**Figure 4:** The selected optical micrographs obtained at *t_c2_* = 15 min and *T_c_* = 135 °C after fiber pulling with different pulling distances. (**a**) 125 μm, (**b**) 250 μm, (**c**) 500 μm, (**d**) 750 μm. The fiber-pulling rate was 12.5 μm/s.

**Figure 5:** The structure evolution of the iPP samples during the cooling process from both the structured and supercooled melts. The selected SAXS profiles were derived from the cooling process: (**a**) from the structured melt (partially melted iPP with the thermal history shown in Figure 1) and (**b**) from the supercooled melt; three selected WAXS profiles were shown in (**a**,**b**), as inset, respectively. (**c**) The evolution of invariant *Q* derived from SAXS data and (**d**) crystallinity derived from WAXS data, both from the structured and supercooled melt. The insets in (**c**,**d**) were the evolution of *Q* and crystallinity during the isothermal crystallization at 135 °C, respectively.

The article "Investigation of the Ordered Structure in Partially Melted Isotactic Polypropylene" was retracted in 2023. Reasons: no approval from the institution; copyright claims.

**Figure 6:** The structural evolution of the iPP sample during the heating process. The sample was prepared, with a thermal history as shown in Figure 1. (**a**) The selected SAXS profiles in log-log coordinate and (**b**) the corresponding WAXS profiles that were obtained during the heating process; (**c**) the evolution of one-dimensional electron density correlation function, *K(z)*. The evolution of long-period (*d_ac_*) and lamellae thickness (*d_c_*) were shown as inset; (**d**) the corresponding evolution of crystallinity derived from the WAXS profiles.

**Figure 7:** The SAXS scattering profile of iPP, obtained at 170 °C for a holding time of 10 min. The best fit (solid line) is also shown. The corresponding simultaneous WAXS profile and diagrammatic sketch for cylindrical nanocrystals are shown at the right top and left bottom as inset, respectively.

## Data Availability

The data presented in this study are available within the current manuscript.
